The article "Digital Image Art Style Transfer Algorithm Based on CycleGAN" was published in 2022. Journal: Comput Intell Neurosci.

# Digital Image Art Style Transfer Algorithm Based on CycleGAN

**DOI:** 10.1155/2022/6075398

**Published:** 2022-01-13

**Authors:** Xuhui Fu

**Affiliations:** Culture and Art Management of Hunan University, Korea, Guangzhou City 62399, Republic of Korea

## Abstract

With the continuous development and popularization of artificial intelligence technology in recent years, the field of deep learning has also developed relatively rapidly. The application of deep learning technology has attracted attention in image detection, image recognition, image recoloring, and image artistic style transfer. Some image art style transfer techniques with deep learning as the core are also widely used. This article intends to create an image art style transfer algorithm to quickly realize the image art style transfer based on the generation of confrontation network. The principle of generating a confrontation network is mainly to change the traditional deconvolution operation, by adjusting the image size and then convolving, using the content encoder and style encoder to encode the content and style of the selected image, and by extracting the content and style features. In order to enhance the effect of image artistic style transfer, the image is recognized by using a multi-scale discriminator. The experimental results show that this algorithm is effective and has great application and promotion value.

## 1. Introduction

The specific characteristics of artistic schools are mainly artistic styles, and different styles also present different cultural connotations and backgrounds. Image art style transfer is mainly the processing of digital images, which refers to the method of forming new image features by fusing the features of different images with each other. There are more and more achievements in the field of deep learning. For example, in 2015, scholar Gatys proposed a method of image art style transfer, through image reorganization, segmentation, and other methods, to generate a confrontation network model. It has also become particularly applicable in image processing, which has attracted the attention of many scholars. The main principle is to improve the performance of neural networks through adversarial training. In order to ensure the effectiveness and operability of the network, the applicability of the model is ensured by adjusting the introduction mechanism of the generative confrontation network and adjusting the frame result. This paper proposes a new artistic style based on the generative confrontation network model, through the extraction of image features and the transfer of image artistic styles. This article focuses on how to finally achieve the artistic visual effects that need to be presented based on the generative confrontation network model. Some problems that can be improved are discovered, and then verified by experiments, practical solutions are proposed, which have certain practical application value and important research significance.

## 2. Related Work

Deep neural networks contain one or more hidden layers of neural network structures, which have good generalization capabilities for complex problems. In theory, deep learning networks can fit arbitrary complex functions and show a powerful ability to learn sample features. In deep learning, CNN is the most commonly used deep neural network for processing computer vision tasks. By sharing the convolution kernel, the CNN can process high-dimensional data, and as long as the training parameters are set, the features in the image can be extracted through layered convolution. Therefore, deep neural networks based on CNN are good at learning and extracting the features and special information contained in images, such as texture features, shape features, boundary features, grayscale features, topological features, and relational structures. The extraction and utilization of these features or information make the application of image processing further enriched and expanded.

Different experts and scholars have carried out different researches on image art style transfer processing. Among them, Sun et al. [1]proposed a CNN architecture with two paths, by extracting the object features and textures of the image, respectively. Features realize image style recognition and output image category. Zhao et al. proposed a [2]high-definition image deep learning training algorithm. The method is mainly divided into three steps: (1) break the traditional method of extracting image features, by extracting the image features of high- and low-resolution images, which can greatly save training time; (2) establish a high-resolution deep learning model based on the dictionary model; (3) transform low-resolution images into high-resolution images. Lu et al.[3–5] believed that the current deep learning model can no longer adapt to the aggregation of multiple images, and proposed a multi-image training model based on an improved neural network. Its framework is mainly to integrate the feature extraction and aggregation algorithms so that the image can extract multiple image features. Castillo et al. proposed constructing a model of artistic target transfer, its principle is mainly to carry out artistic transfer and fusion of a single image object. Regarding the artistic style transfer of dynamic video, Ruder et al. improved on the basis of Gatys, Gatys mainly transfers the artistic style of still images, and Ruder proposes to extract the artistic style of the video image, and extract and transfer the artistic style of the entire video. With the continuous extension and development of image processing methods and technologies in recent years, some creative thinking and methods have also been continuously developed. This paper proposes a generative confrontation network model, which encodes the style and content of the image based on the residual network structure and the encoding and decoding structure. The most important part of network decoding is the generative network, which uses the encoded information to generate the image of artistic style transfer, discriminate the network, make the image effect of the generated network better, and the image more vivid and lifelike, thereby improving the transfer effect of the entire image art style [6–10].

## 3. Related Theoretical Methods

### 3.1. The Algorithm Flow of Generating a Confrontation Network

#### 3.1.1. Algorithm Description

GAN is a powerful generative model. The model is mainly composed of two parts; First, the generative model, which is mainly to generate natural and real images as much as possible; second is the discrimination model, which mainly judges the authenticity of the image [11].

#### 3.1.2. GAN Algorithm Flow

The ultimate goal of GAN is to realize the transfer of artistic style by judging model D and generating model G. G and D are generally nonlinear mapping functions, usually in the form of a network structure such as a multilayer perceptron or a convolutional neural network change. Assuming that *P*_g_(*z*) = {*z*(1),…, *z*(*n*)} is a given random noise sample set that obeys a simple distribution, *P*_data_(*x*) = {*x*(1),…,*x*(*n*)} Is the real data sample set, G is the generating network, and D is the discriminant network (Algorithm 1) [8].

#### 3.1.3. CycleGAN Algorithm

CycleGAN can transform two different styles of images, such as the mutual conversion of photos and oil paintings, day and night, spring, summer, autumn, and winter. Assume that *X* and *Y* are data sample sets in two different fields, G is a generator generated from *X* field to *Y* field, F is a generator generated from *Y* field to *X* field, it is to identify the *X* field data (real *X* field sample). The true and false discriminator of the *X* field data is generated by F, and F is a discriminator for authenticating the *Y* field data (real *Y* field samples and *Y* field data generated by G), which is a cycle consistent loss. The CycleGAN algorithm is described as follows (Algorithm 2) [9].

### 3.2. Image Art Style Transfer Method

The essence of the image to image conversion task is to learn the mapping between *X* and *Y* image domains: *G*_*XY:*_*X* ⟶  *Y* and *G*_*YX*_: *Y* ⟶ *X*. The goal of the unsupervised translation is to restore this mapping using unpaired samples in the original data. This method combines the instance information and adds a set of instance attribute information to the original image *x* to improve the image to image translation effect. Therefore, this method can be understood as learning *X* × *A* and *Y*  × for the joint mapping between B, each network is designed to simultaneously encode the image and the corresponding instance mask. The method is described in detail as follows:

CycleGAN is selected as the basic structure, and the periodic consistency loss is used to encourage *G*_*YX*_ (*G*_*YX*_(*x*)) ≈ *x* and G_*XY*_ (G_*YX*_ (*y*) ≈ *y*. As shown in Figure 1, it is composed of two generators *g* and F, and two discriminators *D*_Y_ and *D*_X_. It is assumed that the given source image data set and target image data set are {*x*_*i*_}_*i*=1_^*N*^ ∈ *X*  and {*y*_*i*_}_*j*=1_^*M*^ ∈ *Y* , N and *M* represent the data set size of the source image and the target image, respectively, *X*_i_ represents the first image in the source image, and *y*_j_ represents the j^th^ image in the target image.

The adversary discriminator *D*_Y_ is responsible for distinguishing the original image {y} from the generated image {*G*(_*x*_)}, and the adversary discriminator *D*_X_ is also responsible for distinguishing the original image{*x*} from the generated image {*F*_(*y*)_}. This structure is circular, that is, converting from one domain to another and then returning. Among them, generators G and F and discriminators *D*_*Y*_ and *D*_*X*_ follow the structure in Figure 1

For the task of this paper, the structure is also maintained, and the whole includes two generators G_XY_ and G_YX_, as well as the corresponding adversary discriminators *D*_Y_ and *D*_X_. First train the generator *G*_*XY*_: *X* × *A* ⟶ *Y*, which simultaneously encodes and converts the original data (*x*, *a*) to the target domain data *y*′. The generator first inputs the original photo and the corresponding segmentation mask, then uses the image feature extractor to extract features from the photo and mask, respectively, connects the corresponding image with the mask features, feeds them back to the image generator, and finally outputs the transformed image. The adversary discriminator *D*_Y_ : *Y* × *B* (“*Y*,” “not *Y*”}, where dy encodes *y* and *b* (or *y*′ and *b*′) at the same time and then determines whether the data is in the target domain *Y* × *B*. The results are fed back to the generator or discriminator to be improved. The specific structure is shown in Figure 2.

For generator G_YX_ : *Y* × *B* ⟶ *X*, which simultaneously encodes and converts the original data (*y*′, *b*′) to the target domain data X. The generator first inputs the photo generated by *G*_*XY*_ and its corresponding segmentation mask, then uses the image feature extractor to extract features from the photo and mask, respectively, connects the corresponding image with the mask features, feeds them back to the image generator, and finally outputs the transformed image. The adversary discriminator *D*_X_ : *X* × *A* (“x,” “not *X*”}, where DX encodes x′ and a (or *x* and *a*) at the same time, then distinguish whether the data is in the target domain *X*×*A*, and feedback the results to the generator or discriminator to be promoted. The specific structure is shown in Figure 3.

Through the continuous game and learning using the generator and discriminator, the generator can finally generate an image with the style of the target area, while keeping the background and corresponding structure position completely consistent with the original image. For our task, input the image containing the target clothing and the segmentation mask corresponding to the target clothing. After the whole model generation process, we can finally fix the clothing style migration task in the specific area of the target clothing, that is, complete the corresponding style migration of the target clothing while keeping the content and style of other areas unchanged. In addition, according to the target task requirements of this paper, the corresponding mask should be completely consistent before and after the image conversion, that is, the mask of the same image input generator should be the same as that in the discriminator in the whole process, which can be expressed as *a* = *b*′.

## 4. Image Art Style Transfer Based on Generative Confrontation Network

This article mainly improves the CycleGAN network to realize the artistic style transfer of images. Through the improvement of the CycleGAN network, the effect of image art style transfer is improved on the premise of reducing the calculation resources and calculation time occupied by the algorithm. Partial optimizations have been made in all aspects of training for research purposes. This chapter will sequentially introduce the image art style transfer network design based on the generative confrontation network, the design of the loss function, the training process and testing process of the network, the experimental environment, and the analysis of the experimental results [12–14].

### 4.1. Image Art Style Transfer Network Design Based on Generative Confrontation Network

#### 4.1.1. Encoder Design

*(1) Content Coding*. The new content encoder in the network structure of this article adopts the autoencoder network model. The autoencoder uses a neural network architecture. In the self-encoder, the network part from the input layer to the coding layer is called the encoder, and the network part from the coding layer to the output layer is called the decoder [15].

The content encoder in the network structure of this article is mainly composed of the residual network. In 2016, He et al. suggested residual learning in the framework of ResNet, the input of the residual network is *x*, which is added to the output *F*(*x*) of the function through the shortcut operation, and the output is *F*(*x*) and *x F*(*x*) + *x*. The shortcut connection in the residual network increases the number of layers of the network, makes the extracted image features richer, and can effectively avoid the gradient disappearance and gradient explosion of the network [16]. The deep residual network can be effectively applied to the fields of image classification, image target detection, and image target localization. The content encoder in this article mainly uses an improved residual network, adding an instance normalization layer and a regular activation function after the convolutional layer. The schematic diagram of the residual structural unit in the content encoder is shown in Figure 4.

The network structure diagram of the content encoder is shown in Figure 5.

The specific process of the content encoder is described as follows:

1. The input picture is a 256 × 256 pixel three-channel image, which is down-sampled; the first layer uses a 7 × 7 size convolution kernel, the number of convolution kernels is 64, the sliding step is 1, and the filling size is 3, then the instance normalization process is performed, and finally, the ReLU activation process is performed.
2. The second and third layers both use 4 × 4 convolution kernels, the number of convolution kernels is 128 and 256, respectively, the sliding step size is 2 for both layers, and the filling size is 1, and then the instance is normalized, and finally the ReLU activation processing is carried out.
3. Then use 2 residual modules, there are two convolutional layers in the residual module, the number of convolution kernels in each convolutional layer is 256, the size of the convolution kernel is 3 × 3, and the sliding step size is 1 for all, the padding size is 1, then the instance normalization process is performed, and finally the ReLU activation process is performed; specifics are as shown in Table 1.

*(2) Style Coding*. The new style encoder in the network structure of this paper adopts the variational autoencoder network model. Variational autoencoders require the hidden vectors generated by encoding to follow a Gaussian distribution. This restriction enables the encoder to understand the underlying laws of the training data and enables the encoder to learn the hidden variable model of the input data. The ordinary autoencoder learns a certain function through training data, and the variational autoencoder can learn the probability distribution of the parameters based on the training data. The style encoding of the image adopts a variational autoencoder to increase the randomness of style features [17].

The specific implementation method of the variational autoencoder is to change the output result of the encoder from one to two in the encoding stage, and the two vectors correspond to the mean vector and the standard deviation vector. and the hidden code vector is obtained by random sampling of the probability model [18–20].

The variational autoencoder can form a hidden vector of Gaussian distribution, randomly sample a hidden encoding vector from the Gaussian distribution as the style feature of the image, and then input the extracted style feature into the generation network. The network structure diagram of the style encoder is shown in Figure 6.

The specific process of the style encoder is described as follows:

1. The input picture is a 256 × 256 pixel three-channel image, which is down-sampled; the first layer uses a 7 × 7 convolution kernel, the number of convolution kernels is 64, the sliding step is 1, and the filling size is 3, then proceed to the ReLU activation reason.
2. The second to fifth layers all use 4 × 4 convolution kernels, the number of convolution kernels are 128, 256, 256, 256, respectively, the sliding step size is 2, the padding size is 1, and the ReLU activation processing is performed; then the average pooling operation is carried out.
3. The last layer uses a 1 × 1 size convolution kernel to realize the function of full connection. The number of convolution kernels is 8, the sliding step is 1, no padding, and no activation function; specifics are as shown in Table 2.

#### 4.1.2. Generating Network Design

This article improves the generation network. In the process of implementing the image art style migration of the CycleGAN network, the generation network uses the U-net jump cascade network structure. The U-net performs multiple splicing in the decoding part and the encoding part, not only the previous decoding The result is used as input and the corresponding encoding part is also used as input for decoding so that the detailed information and high-level semantic information of the input image can be retained, but the U-net network structure occupies a large amount of memory, which increases the number of network calculations and the generated image. The result of artistic style transfer is rather vague [21–23]. In this paper, the generation network mainly uses the residual network structure, and at the same time, the improved generation networks G1 and G2 have the same network structure, but the purpose is different. The purpose of generating the network G1 is to receive the content and style features of the image, and then through the calculation of the intermediate hidden layer, so that the content of the image after the artistic style transfer remains unchanged, which improves the robustness of the network and makes the generated image more realistic. The generation network is a fully convolutional network, which uses residual structural units, up-sampling, and convolution operations to complete the artistic style transfer of the image. The residual structural unit used in the generation network is different from the residual structural unit used in the content encoder.

The normalization method of the residual structural unit in the network uses adaptive normalization. The adaptive normalization method can speed up the stylization of the image and make the generated image retain a strong style. In the generation network, the content information and style information is first input into the residual network at the same time, and after 4 residual module units, specifics are as shown in Figure 7.

The generative network is a convolutional neural network. The input is style features and content features, and the output is an image after artistic style transfer. The specific process is described as follows:

1. The input style coding and content coding first go through 4 residual network structures, in which each residual network structure uses a 3 × 3 size convolution kernel, the number of convolution kernels is 256, the sliding step size is 1, the padding size is 1, the normalization method uses adaptive normalization, and then performs the ReLU activation processing.
2. Use the nearest neighbor interpolation to double the size of the image, and then uses a 5 × 5 size convolution kernel. The number of convolution kernels are 128, 64, sliding step lengths are 1 for both, the padding size is 2, and the normalization method uses layer normalization, and then performs the ReLU activation processing.
3. The last layer uses a 7 × 7 convolution kernel, the number of convolution kernels is 3, the sliding step size is 1, and the padding size is 3. Then perform Tanh activation function processing and output the image after the artistic style transfer. Specifics are as shown in Table 3.

As a result of artistic style transfer, some grid-like images often appear. This is because the images of artistic style transfer are generally low-scoring and have high-level semantic information. After the features of the image are extracted through the convolutional neural network, the features are combined to complete the artistic style transfer of the image.

#### 4.1.3. Discriminant Network Design

The discriminant network in the CycleGAN network uses a convolutional neural network to extract the features of the entire image and then based on the extraction to distinguish the features. However, this method is easy to ignore the detailed information of the image, resulting in problems such as blurring and loss of details in the generated image. This paper uses the multiscale discriminant network structure in the construction of the discriminant network. The multiscale discriminant network structure is an improvement of the block discriminant network structure. The block discrimination network structure is to discriminate image blocks, and finally, take the average value as the final discrimination result of the discrimination network. Compared with discriminating the entire image, the block discrimination network makes the generated image closer to reality.

The multiscale discriminant network combines multiple block discriminant networks to enhance the discriminative ability of the discriminant network. In this way, this article promotes the generated images to be more realistic, thereby improving the quality of the generated images.

It is judged that the network structure of networks D1 and D2 is the same. In order to accelerate the convergence speed of the network and improve the generalization performance of the model, to make the image of the artistic style transfer more lifelike, the multiscale discriminator used in this article is composed of two identical discriminators, and each discriminator model has the same network structure. Discrimination, using the discriminant results of image blocks of different sizes as the final output, thereby improving the discriminative ability of the discriminant network. The discriminant network used in this paper is shown in Figure 8.

In the final analysis, the discriminant network is a convolutional neural network composed of a convolutional layer and a fully connected layer. The main principle is to compare and analyze the features of the sample images. The specific structure diagram is shown in Figure 9.

The network structure of the discriminant network consists of 4 convolutional layers and 1 fully connected layer. The specific process is described as follows:

1. The input image is a three-channel image with a size of 256 × 256.
2. The first to fourth layers all use 4 × 4 convolution kernels, the number of convolution kernels are 64, 128, 256, and 512, the sliding step size is 2 for both, the filling size is 1, and the LReLU activation process is performed.
3. The fifth layer uses a 1 × 1 convolution kernel, the number of convolution kernels is 1, and the sliding step is 1, specifics are as shown in Table 4.

As shown in Table 4, in order to prevent the problem of gradient disappearance during the training process of the generative adversarial network, this paper uses the LReLU activation function in the activation function of the discriminant network except for the output layer. The last layer uses a 1×1 size convolution kernel to realize the function of full connection, convert multi-dimensional input data into one-dimensional, and output the discriminant result of the discriminant network.

### 4.2. Design of Loss Function

The CycleGAN total loss consists of three parts: two adversarial losses and a cycle consistent loss. Taking *x*⟶G(*x*)⟶F(G(*x*)) as an example, the *x* ⟶ *G*(*x*) adversarial loss is

(1) $$\begin{array}{c} l_{GAN}\left(G,D_{y}\right)=E_{y∼pdata\left(y\right)}\left[\log\;D_{y}\left(y\right)\right]+E_{x∼pdata\left(x\right)}\left[\log\left(1-D\left(G\left(z^{\left(i\right)}\right)\right)\right)\right]. \end{array}$$

The confrontation loss of *G*(*x*) ⟶ *F*(*G*(*x*)) is

In the training process of the network, the loss function can speed up the training of the network and improve the quality of image art style transfer.

## 5. Experiment and Result Analysis

### 5.1. Experimental Environment

The article mainly uses Python to write the source code for generating the confrontation network model. The entire deep learning framework is mainly implemented by TensorFlow. The example chosen this time is to migrate the artistic style of different images in summer and winter. The database is summer2winter_yosemite. The entire database has 4482 photos in summer and winter. The training set divides the photos into two folders trainA and trainB according to 8 : 2; the test set is divided into testA folders and testB folders. In the experiment, the batch size is set to 1, and the epoch is set to 10. Through repeated iterations, the Adam optimization parameters learning rate is set to 0.001 for optimization [24].

In the experiment established in this paper, the parameters of the image reconstruction loss function and the content encoding loss function are set, respectively. The weight of the image reconstruction loss function *λ*_x_ is set to 10.0, the weight *λ*_c_ of the content encoding loss function is set to 1.0, and the cyclic consistency loss weight of the function *λ*_cyc_ is set to 10.0, and the counter loss function *λ*_gan_ is set to 1.0, as shown in Table 5.

### 5.2. Experimental Results and Analysis

In the process of running the model, you need to save the encoder, generate a network, discriminant network parameter settings, and model running parameter settings in a file every 30 times of training. When the training is interrupted due to external factors, the model has a memory function, and it can continue to run from the interrupted position until the training is completed. After all network training is completed, the artistic style is transferred through the saved model file information.  Figure 10 is the winter image after the summer image migration experimental results of artistic style photos.

After testing the image art style migration of the summer2winter_yosemite dataset, it can be seen from Figure 10 that the algorithm model established in this paper realizes the conversion and fusion of summer and winter image styles, and the converted images can also match The experimental results of the summer and winter images in the dataset.

## 6. Conclusion

Image art transfer technology has now been widely used and developed prospects, and has relatively successful cases in many fields, but also attracts a large number of experts and scholars to study. This paper proposes an improved generative adversarial network model, which improves the traditional drawbacks of artistic style transfer due to blurred images. The method can extract the content and style characteristics of the selected data set images at the same time. Based on the predecessors, the traditional generative confrontation network model is improved. The content and style encoder of the model are used to extract the features of the image under study. The automatic encoder based on the neural network applies the normalization method to the content and style features. Fusion changes the deconvolution operation in the traditional CycleGAN network, uses image size and convolution, improves the traditional discriminant network, and uses multiscale discriminators to further improve the overall effect of artistic style fusion and migration.

## Figures and Tables

**Figure 1:** Periodic consistent generation countermeasure network model.

**Figure 2:** Generator and discriminator model 1.

**Figure 3:** Generator and discriminator model 2 as a whole.

**Figure 4:** Residual structure unit in the content encoder.

**Figure 5:** Content encoder structure diagram.

**Figure 6:** Structure diagram of style encoder.

**Figure 7:** Generate network structure diagram.

**Figure 8:** Discrimination network.

**Figure 9:** Discrimination network structure diagram.

**Figure 10:** Summer to winter experiment. (a) Original image. (b) Image after artistic style transfer. (c) Original image. (d) Image after artistic style transfer.

**Algorithm 1:** GAN algorithm.

**Algorithm 2:** CycleGAN algorithm.

**Table 1:** Network information table of content encoder.

Operate	Kernel	Strides	Padding	Norm	Activation
Conv	(7,7,64)	1	3	Instance_Norm	ReLU
Conv	(4,4,128)	2	1	Instance_Norm	ReLU
Conv	(4,4,256)	2	1	Instance_Norm	ReLU
Resblock1	(3,3,256)	1	1	Instance_Norm	ReLU
Resblock2	(3,3,256)	1	1	Instance_Norm	ReLU

**Table 2:** Style encoder network information table.

	Kernel	Strides	Padding	Activation
Conv	(7,7,64)	1	3	ReLU
Conv	(4,4,128)	2	1	ReLU
Conv	(4,4,256)	2	1	ReLU
Conv	(4,4,256)	2	1	ReLU
Conv	(4,4,256)	2	1	ReLU
Pooling	—	—	—	—
Fc	(1,1,8)	1	—	—

**Table 3:** Generate network information table.

Operate	Kernel	Strides	Padding	Norm	Activation
Resblock1	(3,3,256)	1	1	Adaptive_Instance_Norm	ReLU
Resblock2	(3,3,256)	1	1	Adaptive_Instance_Norm	ReLU
Resblock3	(3,3,256)	1	1	Adaptive_Instance_Norm	ReLU
Resblock4	(3,3,256)	1	1	Adaptive_Instance_Norm	ReLU
up_Sample	—	—	—	—	—
Conv	(5,5,128)	1	2	Layer_Norm	ReLU
up_Sample	—	—	—	—	—
Conv	(5,5,64)	1	2	Layer_Norm	ReLU
Conv	(7,7,3)	1	3	—	Tanh

**Table 4:** Discrimination network information table.

Convolution number	Kernel	Strides	Padding	Activation
Conv	(4,4,64)	2	1	LReLU
Conv	(4,4,128)	2	1	LReLU
Conv	(4,4,256)	2	1	LReLU
Conv	(4,4,512)	2	1	LReLU
Fc	(1,1,1)	1	—	—

**Table 5:** Loss function weight settings.

Parameter	value
*λ*_*x*_	10
*λ*_*c*_	1
*λ*_*s*_	1
*λ*_gan_	1
*λ*_cyc_	10

## Data Availability

The dataset can be accessed upon request.
